# Detection and differentiation of *Borrelia burgdorferi *sensu lato in ticks collected from sheep and cattle in China

This article has been retracted.

**DOI:** 10.1186/1746-6148-7-17

**Published:** 2011-04-29

**Authors:** Qingli Niu, Guiquan Guan, Jifei Yang, Yuguang Fu, Zongke Xu, Youquan Li, Miling Ma, Zhijie Liu, Junlong Liu, Aihong Liu, Qiaoyun Ren, Wayne Jorgensen, Jianxun Luo, Hong Yin

**Affiliations:** 1 State Key Laboratory of Veterinary Etiological Biology, Key Laboratory of Veterinary Parasitology of Gansu Province, Key Laboratory of Grazing Animal Diseases MOA, Lanzhou Veterinary Research Institute, Chinese Academy of Agricultural Sciences, Lanzhou 730046, China; 2 Centre of Animal Science, QAAFI, University of Queensland 4072 Australia

## Abstract

**Background:**

Lyme disease caused by *Borrelia burgdorferi *sensu lato complex is an important endemic zoonosis whose distribution is closely related to the main ixodid tick vectors. In China, isolated cases of Lyme disease infection of humans have been reported in 29 provinces. Ticks, especially ixodid ticks are abundant and a wide arrange of *Borrelia *natural reservoirs are present. In this study, we developed a reverse line blot (RLB) to identify *Borrelia *spp. in ticks collected from sheep and cattle in 7 Provinces covering the main extensive livestock regions in China.

**Results:**

Four species-specific RLB oligonucleotide probes were deduced from the spacer region between the 5S-23S rRNA gene, along with an oligonucleotide probe which was common to all. The species specific probes were shown to discriminate between four genomic groups of *B. burgdorferi *sensu lato i.e. *B. burgdorferi *sensu stricto, *B. garinii, B. afzelii*, and *B. valaisiana*, and to bind only to their respective target sequences, with no cross reaction to non target DNA. Furthermore, the RLB could detect between 0.1 pg and 1 pg of *Borrelia *DNA.

A total of 723 tick samples (*Haemaphysalis, Boophilus, Rhipicephalus *and *Dermacentor*) from sheep and cattle were examined with RLB, and a subset of 667 corresponding samples were examined with PCR as a comparison. The overall infection rate detected with RLB was higher than that of the PCR test.

The infection rate of *B. burgdoreri *sensu stricto was 40% in south areas; while the *B. garinii infection rate *was 40% in north areas. The highest detection rates of *B. afzelii *and *B. valaisiana *were 28% and 22%, respectively. Mixed infections were also found in 7% of the ticks analyzed, mainly in the North. The proportion of *B. garinii *genotype in ticks was overall highest at 34% in the whole investigation area.

**Conclusion:**

In this study, the RLB assay was used to detect *B. burgdorferi *sensu lato in ticks collected from sheep and cattle in China. The results showed that *B. burdorferi senso stricto *and *B. afzelii *were mainly distributed in the South; while *B. garinii *and *B. valaisiana *were dominant in the North. *Borrelia *spirochaetes were detected in *Rhipicephalus *spp for the first time. It is suggested that the *Rhipicephalus *spps might play a role in transmitting *Borrelia *spirochaetes.

## Background

Lyme borreliosis has been recognized as the one of most common vector-borne diseases in the world. The disease was first reported in the USA by Steere in 1975. Subsequently its clinical manifestations were described by a scholar in Yale University in 1977, and named Lyme disease in 1980 [1]. Burgdorfer and his colleagues isolated a spirochete and confirmed it as the causative agent of Lyme disease [2]. The spirochaete was formally named *Borrelia burgdorferi *in 1984 [3].

Lyme disease is distributed in over 30 countries and regions of Asia, Europe, America, Africa and Oceania, with more than 0.3 million clinical cases per year [4]. In the USA, it is particularly severe with approximately 20-100 cases per 100,000 [5]. The number of cases is increasing, and the disease was listed as a key target for prevention and control by WHO in 1992 [6].

In China, the disease was first identified in the forest regions of Hailin county in Heilongjiang province in 1986 [7]. Liang and Zhang latter confirmed that three *B. burgdorferi *isolates from the region caused Lyme disease [8]. To date, serological investigations have confirmed that Lyme disease is present in more than 29 provinces and autonomous regions, and more than 130 isolates of *B. burgdorferi *have been recovered from patients, ticks or animals in 19 provinces and autonomous regions [9,10], especially in the northeast forest areas. The prevalence of Lyme disease correlates with the geographic distribution and activity of vector ticks [11]. Of the 109 species of ticks identified in China, Lyme disease pathogens have been isolated from 9 Ixodid ticks, including *Ixodes persulcatus, I. granulatus, I. acutitarsus, H. longicornis, H. bispinosa, H. concinna, H. formosensis, Boophilus microplus *and *Dermacentor silvarum*[12].

The *B. burgdorferi *sensu lato complex comprises at least 13 species, *B. burgdorferi *sensu stricto, *B. garinii, B. afzelii, B. lusitaniae, B. valaisiana, B. bissettii, B. andersonii, B. japonica, B. tanukii, B. turdi, B. sinica, B. spielmanii *and *B. californiensis*. The following five species of *B. burgdorferi *have been isolated from ticks: *B. burgdorferi *sensu stricto (*I. scapularis, I. dammini, I. ricinus *and *I. pacificus*), *B. garinii *(*I. ricinus *and *I. persulcatus*), *B. afzelii *(*I. ricinus *and *I. persulcatus*), *B. lusitaniae *(*I. ricinus*) and *B. valaisiana *(*I. ricinus and I. columnae*) [13-17].

In this study, we developed a reverse line blot (RLB) to detect and differentiate 4 *B. burgdorferi *sensu lato species on the basis of the variable spacer region regions between 5S and 23S rRNA genes sequences. We then used the RLB to investigate the distribution and prevalence of *B. burgdorferi *sensu lato in China.

## Results

### Specificity of the RLB

Amplification of the 5S-23S rRNA gene internal transcribed spacer was performed by nested PCR on four isolates (Figure 1.). The primers specifically amplified the spacer region between 5S-23SrRNA genes sequence from *Borrelia *and no cross-reaction occurred with DNAs from *M. pneumoniae, C. psittasi, Anaplasma. marginale *and *A. ovis*. All probes bound to their respective target sequence only; no cross reaction was observed at dilutions used, resulting in the clear recognition of individual strains, species, or groups. Each of the 4 *B. burgdorferi *species was identified by one of the oligonucleotide probes (Table 1). Isolate BO23 was identified by two oligonucleotide probes: Sl (453-430), and a specific probe recognizing Af (305-278), isolate B31 was identified by two oligonucleotides probes: the Sl (453-430), and a specific probe recognizing Ss (322-299). Isolates SZ, T25, PBr, 20047, IP90 and TN were recognized by two oligonucleotides as well: Sl (453-430), and a specific probe recognizing Ga (322-298). Isolate VS116 was identified by two oligonucleotide probes: Sl (453-430), and a specific probe recognizing Vs (303-278), No signal was detected from genomic DNA of *M. pneumoniae, C. psittasi, A. marginale *and *A. ovis*, or water (Figure 2).

**Figure 1:** **The second PCR amplification of the 5S-23S intergenic spacer region**. Lanes 1-14:BO23: *Borrelia. afzelii*; B31: *Borrelia.burgdorferi *sensu stricto; SZ, T25, PBr, 20047, IP90, TN: *Borrelia. garinii*;VS116: *Borrelia. valaisiana*; *Mycoplasma ovipneumoniane,, Chlamydia psittacii, Anaplasma marginale, Anaplasma ovis *and pathogen-free tick DNA as negative controls.

**Table 1:** Species and their recognition pattern by oligonuclotide probes

Isolate designation	Species	Oligonucleotide*	
		
		Species-specific	Group-specific
BO23	*B. afzelii*	**Af**	
B31	*B. burgdorferi s.s.*	**Ss**	
T25	*B. garinii*		
PBr	*B. garinii*		
SZ	*B. garinii*	**Ga**	**Sl**
20047	*B. garinii*		
IP90	*B. garinii*		
TN	*B. garinii*		
VS116	*B. valaisiana*	**Vs**	

*See Table 3 for oligonucleotide sequence data.

**Figure 2:** **Reverse line blot (RLB) assay specificity test for *Borrelia burgdorferi***. Sl: Probe of *Borrelia burgdorferi *sensu lato; Ga: Probe of *Borrelia.garinii*; Ss: Probe of *Borrelia.burgdorferi *sensu stricto; Af: Probe of *Borrelia. afzelii*;Vs: Probe of *Borrelia. valaisiana*; row 1-14: BO23: *Borrelia. afzelii*; B31: *Borrelia.burgdorferi *sensu stricto; SZ, T25, PBr, 20047, IP90, TN: *Borrelia. garinii*;VS116: *Borrelia. valaisiana*; *Mycoplasma ovipneumoniane, Chlamydia psittacii infections, Anaplasma marginale, Anaplasma ovis *and pathogen-free tick DNA as negative control.

### Comparison of sensitivity of nested PCR and RLB

Sensitivity of the RLB was assessed using 10 fold diluted genomic DNA (10^-1^~10^-12^) of *B. burgdorferi *sensu stricto, *B. garinii, B. afzelii*, and *B. valaisiana*. The RLB system was capable of detecting 1pg of *B. burgdorferi *sensu stricto, *B. afzelii*, DNA and 0.1pg of *B. garinii, B. valaisiana *DNA. The detection level of the nested PCR carried out in parallel was also restricted to about 1pg~0.1pg (Figure 3). Unlike the nested PCR, the RLB was able to identify which species *B. burgdorferi *sensu stricto, *B. garinii *or *B. afzelii*, the tick was infected with.

**Figure 3:** **The sensitivity of the RLB assay for B. burgdorferi sensu lato**. Plate 1 shows the sensitivity of the nested-PCR using Ba and Bb probes; Plate 2 shows the sensitivity of RLB using Ba and Bb probes; Plate 3 shows the sensitivity of the nest-PCR using Bg and Bv probes; Plate 4 shows the sensitivity of the RLB of using Bg and Bv probes. Lane1-12: 10^0-11 ^10 × fold dilution DNA of Genome for B.burgdorferi sensu lato Row 1-6: oligonucleotide probe of B. burgdorferi sensu lato (Sl); oligonucleotide probe of B. burgdorferi sensustricto; (Ss); oligonucleotide probe of B. garinii( Ga); oligonucleotide probe of B. afzelii (Af); oligonucleotide probe of B. valaisiana (Vs); oligonucleotide probe of B. burgdorferi sensu lato (Sl).

### Detection of *B. burgdorferi *sensu lato in ticks collected from sheep and cattle in China

The prevalence of each *B. burgdorferi *species was identified by RLB and PCR (Table 2). The number of samples in which *B. burgdorferi *sensu stricto, *B. garinii, B. afzelii*, or *B. valaisiana *alone were detected were 201 (28%), 245 (34%), 160 (22%), 85 (12%) respectively (Table 2), and 7% (50/723) were mixed infections and mainly in northern China. For the positive samples from southern China, it was found that the majority (40%) of them were infected with *B. burgdorfei *sensu stricto, while *B. garinii *was dominant (40%) in the positive samples from northern China. The results have revealed that most of the positive samples were infected by *B. burgdorfei *sensu stricto, *B. garinii *and/or *B. afzelii*. Sixty-nine samples (Shangzhi and Huichun), 15 samples (Lintan) and 1 sample (Huaihua) were detected from *Dermacentor, Haemaphysalis *and *Boophilus*, which belonged to *B. valaisiana*.

**Table 2:** Comparison of the results of examination of field tick samples by RLB and PCR

Origin	Genra of tick	No. of tick infected/examined					
		
		RLB					PCR
		
		BB	BG	BA	BV	Mix^a^	
Huaihua	*Boophilus*	62/146(42)	54/146(37)	33/146(23)	1/146(0.7)		44/146(30)
Nanping	*Haemaphysali*	3/39(7.6)	16/39(41)	1/39(2.6)			1/39(2.6)
Huizhou	*Rhipicephalus*	4/48(8.3)	7/48(14.6)	3/48(6.3)			14/45(31)
Laibin	*Boophilus*	41/42(98)	3/42(7)	41/42(98)			15/39(38)
**Total in south**		110/275(40)	80/275(29)	78/275(28)	1/275(0.4)		74/269(27)
Shangzhi	*Dermacentor*	44/154(29)	91/154(59)	44/154(29)	54/154(35)	33/154(21)	7/134(5)
Huichun	*Dermacentor*	24/160(15)	34/160(21)	16/160(10)	15/160(9.4)	9/160(5.6)	3/130(2.3)
**Total in Northeast**		68/314(22)	125/314(40)	60/314(19)	69/314(22)	42/314(13)	10/264(4)
Lintan	*Haemaphysalis*	23/134(17)	43/134(32)	22/134(16)	15/134(11)	8/134(6)	10/134(7)
**Total**		201/723(28)	248/723(34)	160/723(22)	85/723(12)	50/723(7)	94/667(14)

^**a**^**BB**: *B. burgdorferi *sensu stricto, **BG**: *B. garinii***, BA**: *B. afzelii*, **BV**: *B. valaisiana*

**Mix**: a tick is infected by more than one species of *B. burgdorferi*.

## Discussion

Lyme disease is a tick-borne disease caused by *Borrelia*. Animals such as cattle, sheep, horses, dogs and rats can be infected by the pathogen, and in most cases, play a role as reservoirs with varied clinical symptoms [18-20]. Lyme disease spirochetes have been isolated and detected from the following tick vectors: *Ixodes persulcatus, I. crenulatus, Haemaphysalis longicornis, H. japonica, Boophilus microplus, Dermacentor silvarum *and *D. nuttalli *[21]. The main mode of transmission is via the salivary gland when infected ticks feed on mammalian hosts. The infection rate of *I. persulcatus, I. granulates *and *H. bispinosa *were 40%-50%, 16%-40% and 24% respectively in north of China, suggesting that *I. persulcatus *is the principal vector of Lyme disease spirochete in northern China, while *I. granulates *and *H. bispinosa *are the main vectors in the south of China [22].

Although Lyme disease was found more than 20 years ago in China, knowledge of the epidemiology of the causative organism in the tick vectors is limited. We therefore considered that it would be very useful to develop a validated method to detect all four Lyme disease pathogens associated with ticks to better understand the epidemiology of the disease in different regions of China.

The RLB assay was here developed into a useful diagnostic tool to simultaneously detect and differentiate *B. burgdorferi *subspecies in ticks. Each species can be identified by a species-specific oligonucleotide probe using a line-blotter apparatus which is quickly becoming a standard molecular tool for diagnostic and epidemiological studies in an increasing number of laboratories all over the world. In this study, a RLB assay was established based on the spacer region between 5S and 23S rRNA genes of *B. burgdorferi senso lato*. *B. burgdorferi *sensu stricto, *B garinii, B. afzelii*, and *B. valaisiana *as decribed Barandika et al [23]. All four *Borrelia *species could be differentiated with 4 species-specific oligonucleotides while the oligonucleotide probe Sl designed specifically for the genera of *B. burgdorferi *hybridized with all 4 species. Any new species or genotype that may present would therefore be detected by the SI probe but not by the species-specific probes. Meanwhile, in order to confirm whether there was false positives, the sequence analysis of 120 samples was conducted for amplicons (PCR product) from these samples by random sampling. In all cases, it was found that the fragment was about 400 bp and 250bp, and the homology was 99.5% and 99.2% with the 5S-23S rRNA intergenic spacer region gene of *B. burgdorferi *by DNAstar analysis, suggesting that the ticks were infected by *B. burgdorferi *sensu lato. The RLB was a reliable diagnostic tool and when PCR amplification steps were included, the specificity was further improved. Different strains can be detected concurrently, and coinfection of different strains of *B. burgdorferi *sensu lato could be distinguished.

We have shown here that the infection rate of *Borrelia *spirochaetes in ticks varies considerably between different geographical regions. *B. burgdorferi *sensu stricto is found more frequently in the South (Laibin and Huaihua) and *B. garinii *more frequently in the Northeast (Shangzhi and Huichun) and Northwest (Lintan), this is not accordance with the recent reports [24]. Our results do not agree with previous findings which suggest that *B. afzelii *is the dominant species in northeast China. However, in the present study, the *B. afzelii *infection rate of samples from the north was lower than those samples infected with *B. garinii *and *B. burgdorferi *sensu stricto. Although the infection rate of ticks with *B. afzelii *was 19%, which was much higher than that previously reported [25], the low infection rate of *B. afzelii *might be associated with the limited number of ticks collected from field. Another explanation could be that the tick infection rate of each of the four *Borrelia *varies among samples from different regions, and it is possible that samples in this study were collected from areas where the tick infection rate of *B. afzelii *is lower.

To the best of our knowledge, this is the first study in which Lyme disease species of *B. burgdorferi *sensu lato were detected by RLB in field ticks in China. The prevalence and distribution of *Borrelia *spirochaetes in ticks are key factors for risk assessment of Lyme borreliosis. From our results, it could be seen that *B. garinii *is the dominant species and widely distributed in China, which agrees with the previous data [26-28]. *B. afzelii *and *B. burgdorferi *sensu stricto have been found only in a limited number of ticks, however, the tick infection rate with *B. burgdorferi *sensu stricto was higher than that of *B. afzelii*, which is different from previously reported.

*B. valaisiana *has only been isolated from rats from Guizhou Province in China and it has been assumed that distribution of *B. valaisiana *is confined to the southwest of China [29]. In this study *B. valaisiana *was detected in relatively high levels in the samples from northeast China (Table 2). Masuzawa et al [30] have confirmed that *B. valaisiana *is present in Korea which is geographically very close to northeast China. The prevalence of *B. valaisiana *varied among our study sites. It could be inferred that the distribution of *B. valaisiana *is much wider than originally thought. Previous reports suggested that *B. valaisiana *was more difficult to isolate from clinically diagnosed cases of Lyme Borreliosis than genomospecies *B. burgdorferi *sensu stricto, *B. afzelii *and *B. garinii *[14,31]. As most of the current prevalence data on Lyme disease are from human medical institutions and identification of *Borrelia *is based on the isolation, it is reasonable to believe that in northeast China, *B. valaisiana *is more prevalent but may be misdiagnosed due to the difficulty of isolation of the pathogen.

We collected samples of four genera of ticks from sheep and cattle, which were *Haemaphysalis *(n = 173), *Boophilus *(n = 188), *Rhipicephalus *(n = 48) and *Dermacentor *(n = 314) from seven regions, where the primary forests are preserved. The infection rates of the four genera of ticks with the four species of *Borrelia burgdorferi *l were 15%, 34%, 13% and 0.8% (*Haemaphysalis*), 54%, 28%, 39% and 0.05% (*Boophilus*), 0.8%, 1.4%, 0.6% and 0% (*Rhipicephalus*), and 21%, 39%, 19% and 22% (*Dermacentor*); while the infection rates detected by PCR were 6% (*Haemaphysalis*), 32% (*Boophilus*), 31% (*Rhipicephalus*) and 4% (*Dermacentor*) [31]. Recently, Richter and Matuschka (2010) have found that although about a quarter of *I. ricinus *ticks questing on the pasture were infected by spirochetes, the positive rate of the ticks collected from goats and cattle was much lower, and no molted ticks that had previously engorged or repletion on ruminant harbored Lyme disease spirochetes [32]. The authors also concluded that the spirochetes are cleared from *I. ricinus *ticks during feeding on ruminants. To confirm this hypothesis, more engorged ticks of these four species should be collected to test the status of spirochete infection of their offspring. In the present study, the results indicated that the positive detection rates of the RLB technique were higher than that by PCR. We further confirmed the sensitivity of the RLB, and the detection results of the infection state of three genera of ticks are also consistent with two methods on the whole, except for the results with *Rhipicephalus*. It has been still unknown yet why the positive rate by PCR was higher than by RLB with the *Rhipicephalus ***s**amples. Our data suggests that the infection rate of different genera of ticks is also variable. However, the differences in infection rates among tick species were not statistically significant, and these differences could be due to geographical and seasonal variations of tick and host populations rather than tick vector competence. Because the ticks were collected from animals which could have been already infected with *Borrelia burgdorferi*, we can therefore only say that these ticks are potential vectors. The data showed the infection rate of *Boophilus *with *Borrelia *was relatively high and this species might play a role in transmission of Lyme diseases [21,33]. As *Boophilus *does not readily attach to humans, it could transmit the pathogen between cattle and perhaps sheep, and these infected animals would become reservoirs for other tick species which will attach to humans. These results are consistent with previous studies and confirm that *Boophilus *plays an important role in Lyme disease transmission amongst livestock. It has been reported that *Haemaphysalis *and *Dermacentor *are the vectors of Lyme disease [27,34] yet *Rhipicephalus *spp. have not previously been confirmed as vectors. In this study, we detected *Borrelia burgdorferi *in *Rhipicephalus *spp suggesting that *Rhipicephalus *spp. might transmit *Borrelia burgdorferi*. In the present study, it was not possible to confirm that these four genera of ticks were capable of transmitting *Borrelia *sporochaetes, and the competence of the ticks as vector will need to be determined by further experimental study.

## Conclusion

This study reports development of a RLB assay that is able to detect 4 species of *B. burgdorferi *sensu lato in field ticks simultaneously. The genomic DNA of *B. burdorferi senso stricto *and *B. afzelii, B. garinii *and *B. valaisiana *have been detected in samples prepared from 4 genera of ticks collected from seven different areas in China. These findings extend the knowledge of the epidemiology of *Borrelia burgdorferi *and its possible transmission by adult ticks in China. RLB is a powerful tool for such epidemiological studies and for further investigation of the association between tick vectors *B. burgdorferi *sensu lato species and clinical manifestations of Lyme disease. It can also be used for screening ticks and can easily be expanded to include additional *Borrelia *species. We also demonstrated that *Rhipicephalus *spps are the potential vectors of *Borrelia burgdorferi*. Several tick species may be involved in the transmission of *Borrelia *in China and the high infection rate suggests that there is a high risk of human infection. Little is known of the epidemiology, diagnosis and control of Lyme borreliosis in livestock, and more research is needed.

## Methods

### *Borrelia *strains and culture

Three *B. burgdorferi *sensu lato strains, *B. burgdorferi *sensu stricto (B31), *B. afzelii *(BO23) were purchased from American Type Culture Collection. *B. garinii *(SZ) was isolated from *Dermacentor *ticks as described by Niu et al. [35]. The spirochaetes were cultured in BSKII medium at 33°C as described previously [18]. DNA of standard *Borrelia *genotypes used in the study was provided by Dr. Fingerle (Nationales Referenzzentrum für Borrelien Max von Pettenkofer-Institut, LMU München) in Germany. The designations and origins of the strains are given in Table 1[34,13,36].

### Control samples

DNA is from four species of bacteria, *Mycoplasma ovipneumoniane, Chlamydia psittacii *infections, *Anaplasma marginale *and *Anaplasma ovis*, were provided by colleagues in Lanzhou Veterinary Research Institute, CAAS and used as negative controls.

DNA from adult *Haemaphysalis qinghaiensis *was also used a control. The ticks were originally collected from sheep, goats and cattle in Lintan county, Gansu province. Prior to DNA extraction, the final generation of ticks was fed on splenectomised sheep to confirm absence of any tick borne pathogens. The examination of the sheep by microscopy and PCR proved that the sheep has not been infected by *Borrelia*. Furthermore, the same DNA was tested by both PCR and RLB, and the results were negative. Therefore, the remaining unfed adult ticks of *H. qinghaiensis *were designated a *Borrelia*-free strain of *H. qinghaiensis*.

### Field samples

From March to August in 2009 (Figure 4), ticks (n = 723) were collected on cattle and sheep from Nanping in Fujian province, Huizhou in Guangdong province, Laibin in Guangxi province, Huaihua in Hunan province, Shangzhi in Heilongjiang province, Huichun in Jilin province and Lintan in Gansu province. Ticks were identified to genus using keys previously described by Deng and Jiang 1991 [37].

**Figure 4:** **Map of China showing the number of ticks examined in each of the seven regions in this study**.

### Tick DNA extraction

Each tick was soaked in 70% ethanol in 15 min, dried, and ground in a separate 1.5 ml Eppendorf tube to avoid cross contamination. The sample was incubated with proteinase K for 2h at 56°C, and then boiled at 100°C for 10 min to inactivate proteinase K. After centrifugation, the supernatant was transferred to a fresh sterile microtube, and DNA was extracted using a Genomic DNA Purifcation Kit (Gentra, USA) according to the manufacturer's instructions.

### Primers and probes

Two pairs of primers were designed from 5S-23S rRNA intergenic spacer region [38,39]. They are: 23SN1 (5'-ACCATAGACTCTTATTACTTTGAC-3' 469-446), 23SC (5'-TAAGCTGACTAATACTAATTACCC-3' 92-115) and 5SCB (5'-biotin-GAGAGTAGGTTATTGCCAGGG-3' 243-263), 23SN2 (5'-ACCATAGACTCTTATTACTTTGACCA-3' 469-444).

Species-specific RLB oligonucleotide probes were deduced from the hypervariable 5S-23S rRNA gene intergenic spacer region (Table 3). All the specific oligonucleotide probes contained a N-(trifluoroacetamidohexyl-cyanoethyl, N, N-diisopropyl phosphoramidite [TFA])-C6 amino linker and were diluted to 10-1,200 pmol/150 μl in 500 mM NaHCO_3 _(pH 8.4) to provide optimal sensitivity and specificity (summarized in Table 4).

**Table 3:** Sequence, concentration and position of specific oligonucleotide probes for *B. burgdorferi *sensu lato

Type of primers and isolate	Oligonucleotide Sequence(5'-3')	Concentration used (pmol)	Position on 5S-23S intergenic spacer region
**23SN1**	ACCATAGACTCTTATTACTTTGAC	50	469-446
**23SC**	TAAGCTGACTAATACTAATTACCC	50	92-115
**5SCB**	biotin-GAGAGTAGGTTATTGCCAGGG	50	243-263
**23SN2**	ACCATAGACTCTTATTACTTTGACCA	50	469-444
*B.burgdorfei ***sensu lato (S1)**	a-CTTTGACCATATTTTTATCTTCCA	800	453-430
*B. burgdorferi ***sensu stricto (Ss)**	a-AACACCAATATTTAAAAAACATAA	20	322-299
*B. garinii ***(Ga)**	a-AACATGAACATCTAAAAACATAAA	10	322-298
*B. afzelii ***(Af)**	a-AACATTTAAAAAATAAATTCAAGG	200	305-278
*B. valaisiana ***(Vs)**	a-CATTAAAAAAATATAAAAAATAAATTTAAGG	10	303-278

**Table 4:** Strain designation, species, and geographic origin of isolates used in this study

Strain	Species	Origin	Geographic origin	Reference
BO23	*B. afzelii*	Skin	Germany	13
B31	*B. burgdorferi s.s.*	Ixodes dammini	United States	13
SZ	*B. garinii*	*Dermacentor*	China	35
T25	*B. garinii*	Ixodes ricinus	Germany	13
PBr	*B. garinii*	Human (CSF)	Germany	13
20047	*B. garinii*	I. ricinus	France	36
IP90	*B. garinii*	I. persulcatus	Russia	36
TN	*B. garinii*	Ixodes ricinus	Germany	13
VS116	*B. valaisiana*	Ixodes ricinus	Switzerland	17

### Nested PCR amplification

All DNA samples of ticks and *B. burgdorferi *sensu lato isolates were amplified in duplicate by nested PCR. Genomic DNA of *M. pneumoniae, Chlamydia psittacii, A. marginale *and *A. ovis*, and water were used as controls. Primers, *Taq *DNA polymerase and buffers were obtained from TakaRa (Dalian, China). The first PCR was performed in a reaction volume of 50 μl. For each sample, the PCR mixture was prepared as follows: H_2_O 38.7 μl, 10 × reaction buffer (200 mM Tris-HCl (pH 8.55), 160 mM (NH_4_)_2_SO_4 _and 20 mM MgCl_2_) 5 μl, 10 mM dNTP 4 μl, 50 pmol each of primers 23 SN1 and 23 SC, *Taq *polymerase 1.8 U and 1 μl of DNA sample or water. PCR amplification was performed in an automatic DNA thermocycler (Eppendorf). The program for the first PCR consisted of an initial denaturation at 94°C for 3 min followed by the thermal cycle reaction program of 1 min at 94°C, 90 s at 50°C, and 90 s at 72°C for 40 cycles with a final extension step at 72°C for 5 min. Samples were held at 4°C until analysis. 1 μl of the product from the first PCRs was added to the second PCR tubes containing reaction mixture which were then were briefly vortexed, centrifuged and then transferred to a thermal cycler. After a denaturation step, (1 min at 94°C), 40 rounds of temperature cycling (94°C for 30 s, 55°C for 30 s, and 72°C for 1 min) were performed.

### Analysis of amplified products and sequence analysis

All PCR products were separated electrophoretically in 1.5% agarose and visualized under UV light after ethidium bromide staining.

Nine independent positive clones for each *B. burgdorferi *sensu lato isolates were sequenced using the BigDye Terminator Mix (TaKaRa Company, China). The sequences of the first PCR was size of approximately 362-392 bp, and the second PCR product was 218-235 bp, respectively. The homology was 96.8-98.7% amongst the other isolates in GenBank by DNAstar analysis, confirming that they were from genomic DNA of *Borrelia *species.

### Reverse line blot hybridization

Protocols for preparation of RLB membrane and hybridization were carried out as previously described [40] with the following modifications: Biodyne C membrane was cut into a 14.5 cm square and activated by 10 min incubation in 10 ml freshly prepared 16% (w/v) 1-ethyl-3-(3-dimethylaminopropyl) carbodiimide (EDAC) in demineralized water, in a rolling bottle at room temperature. The membrane was then washed with agitation in demineralized water for 2 min and placed on a supporting cushion in a clean miniblotter system. Each probe was diluted in with water to give a range of concentrations (800 pmol, 400 pmol, 200 pmol, 100 pmol, 50 pmol, 20 pmol and 10 pmol), aliquoted into the miniblotter slot and incubated for 1 min. The solutions were aspirated and the membrane incubated in 100 mM NaOH for 10 min, and then washed at 42°C for 5 min in 2 × SSPE, 0.1% (SDS). Subsequently, the membrane was placed into the miniblotter, perpendicular to its previous orientation. The denatured PCR samples were aliquoted into the slots of the miniblotter for 10 min at 42°C, then aspirated and the membrane washed at 42°C for 10 min in 2 × SSPE, 0.1% SDS. Subsequently, the membrane was treated at 42°C for 45~60 min with peroxidase-labeled streptavidin diluted 1:4,000 in 2 × SSPE/0.1% SDS, washed twice at 42°C for 10 min, and washing twice at room temperature for 5 min in 2 × SSPE, 0.1% SDS. Finally detection of binding was by chemiluminescence performed according to manufacturer's recommendations (Santa Cruz Biotechology ).

### Specificity and sensitivity of the RLB

The RLB was performed by 20 μl of 100ng amplified product of *B. burgdorferi *sensu stricto, *B. garinii, B. afzelii*, and *B. valaisiana *extracted. Meanwhile, *Mycoplasma ovipneumoniane, Chlamydia psittacii, Anaplasma marginale, Anaplasma ovis *and pathogen-free tick DNA as negative control were used as negative controls. The sensitivity of the RLB was tested by hybridizing 20 μl aliquots of 10-fold serially diluted PCR product. The genomic DNA of the four pathogens was serially diluted from 100ng/μl to 0.000001pg/μl by 10-fold dilution as templates for the PCR, and then hybridized by RLB.

## Epidemiological study

A total of 723 ticks were examined by the established RLB assay and the positive and negative samples were recorded to assess the *Borrelia *spirochaetes infection rate in the four genera of ticks. Furthermore, 667 of these same samples were tested with the PCR.

## Authors' contributions

QLN carried out the samples detection, RLB analysis and drafted the manuscript. HY, JXL participated in the design of the study. GQG, JFY, YGF, ZKX, YQL, MLM, JLL, AHL and QYR participated in sampling. WJ reviewed and commented on the manuscript. All authors read and approved the final manuscript.
